The article "MiR-34b inhibits the proliferation and promotes apoptosis in colon cancer cells by targeting Wnt/β-catenin signaling pathway" was retracted in 2024. Reason: duplicated images.

# MiR-34b inhibits the proliferation and promotes apoptosis in colon cancer cells by targeting Wnt/β-catenin signaling pathway

**DOI:** 10.1042/BSR20191799

**Published:** 2019-10-11

**Authors:** Kailun Ye, Chunhua Xu, Tongguan Hui

**Affiliations:** Department of Surgery, First People’s Hospital of Tonglu, Hangzhou 311500, Zhejiang, China

**Keywords:** Colon cancer, Invasion, Migration, MiR-34b, Proliferation, Wnt/β-catenin signaling

## Abstract

Colon cancer is one of the leading cause of cancer deaths that is severely threatening human health. Several microRNAs (miRNAs) have been found to be associated with the tumor genesis of colon cancer. The present study determined the expression of miR-34b in patients with colon cancer and studied the molecular mechanism of miR-34b in the proliferation and apoptosis of human colon cancer Caco-2 cells *in vitro*. In colon cancer patients, the expression of miR-34b was decreased in tumor tissues when compared with the adjacent non-tumor tissues. Furthermore, overexpression of miR-34b inhibited proliferation, migration and invasion, while promoted apoptosis in colon cancer cells. The online bioinformatics sites predicted possible regulatory genes of miR-34b and luciferase reporter assay verify that β-catenin was a direct target of miR-34b. Furthermore, miR-34b overexpression significantly decreased the expression of genes associated with Wnt/β-catenin signaling pathway. In conclusion, our results suggest that miR-34b may inhibit migration and invasion of human colon cancer cells by regulating Wnt/β-catenin signaling and miR-34b may be a key target for the treatment and diagnosis of colon cancer.

## Introduction

Colon cancer remains one of the commonly diagnosed gastrointestinal tumor and it ranks third highest worldwide in terms of cancer-associated mortality rates [1]. It was estimated that approximately 700000 people die from colon cancer and more than 1 million new cases occur each year [2]. Many progressive methods including surgical resection and chemoradiotherapy have been improved for the treatment of colon cancer, while the median survival rate of the disease is still very poor [3]. Therefore, it is urgently necessary to explore molecular mechanisms underlying the pathogenesis of colon cancer since it is helpful for the development of effective therapeutic approaches and new diagnostic markers.

Multiple regulatory factors are involved in the occurrence and development of colon cancer. MicroRNAs (miRNAs) are a class of short non-coding RNA molecules with 19–22 nucleotides in length and they can cause protein degradation through directly binding with target mRNAs [4]. An increasing number of studies have reported that miRNAs play vital roles in modulating multiple malignant cancers by acting as tumor suppressors and oncogenes [5,6]. MiR-34 family, which consists of miR-34a, miR-34b and miR-34c, is thought to be a key mediator in p53 pathway [7,8]. Moreover, miR-34 family is considered to play important roles affecting cancer initiation and progression [9,10]. Previous studies have showed that aberrant expression of miR-34 family may be associated with the proliferation, migration and invasion of colon cancer [11,12]. For example, epigenetic methylation of miR-34a in combination with elevated expression of c-met and β-catenin was observed in colon cancer samples with liver metastases [13,14]. In colon cancer stem cells, miR-34a can regulate cancer stem cell asymmetric division by targeting NUMB and Notch1 [15]. Moreover, a recent study reported that Pien Tze Huang, a traditional Chinese medicine, inhibited the proliferation of colorectal cancer cells by increasing the expression of miR-34c [16]. However, the roles of miR-34b in regulating the migration and invasion of colon cancer cells are still yet to be evaluated.

The article "MiR-34b inhibits the proliferation and promotes apoptosis in colon cancer cells by targeting Wnt/β-catenin signaling pathway" was retracted in 2024. Reason: duplicated images.

In the present study, the expression level of miR-34b in tumor tissues of colon cancer patients was determined. Moreover, the biological roles of miR-34b in the proliferation, migration, invasion and apoptosis of colon cancer Caco-2 cells were examined *in vitro*. We further confirmed that the effects of miR-34b on colon cancer cells might be mediated by the Wnt/β-catenin signaling pathway. These data may provide new insights into the functions of miR-34b in colon cancer progression.

## Materials and methods

### Tissue samples

From August 2016 to September 2018, a total of 27 colon cancer tissues and paired adjacent non-tumor tissues were collected from the patients who underwent surgery in our hospital. All the patients were not treated with chemotherapy or radiotherapy before surgery. Tissue samples were frozen in liquid nitrogen and stored at −80°C until use. This research was approved by the Ethics Committee of our hospital and obtained each patient’s informed consent.

### Cell culture

Human colon cancer cell line Caco-2 was purchased from the Type Culture Collection of the Chinese Academy of Sciences (Shanghai, China). Cells were cultured in a humidified incubator at 37°C in an atmosphere of 95% air and 5% CO_2_, and were maintained in Dulbecco’s modified Eagle’s medium (Gibco, U.S.A.) supplemented with 10% fetal calf serum (Gibco, Australia), 1% non-essential amino acids, 1% sodium pyruvate and 1% penicillin/streptomycin.

### RNA isolation and quantitative real-time PCR

Total RNAs were extracted from tissues and cells by using TRIzol reagent (Invitrogen, U.S.A.) according to the manufacturer’s instructions. The extraction concentration was measured by using a NanoDrop-1000 (Thermo Fisher Scientific, U.S.A.). Synthesis of cDNA was carried out using PrimeScript™ RT Reagent Kit (Takara, China). qPCR was subsequently performed using SYBR® Green PCR Master Mix (Takara, China) with the Applied Biosystems 7900HT real-time PCR machine (Applied Biosystems; Thermo Fisher Scientific, Inc.) following the manufacturer’s protocol. The reaction conditions were as follows: at 95°C for 10 min; 40 cycles at 95°C for 15 s, at 55°C for 30 s and at 72°C for 30 s, and at 72°C for 10 min. Sequences of all primers were listed in Table 1. The relative expression was calculated by the 2^−Δ*C*^t method and each sample was assayed in triplicate.

The article "MiR-34b inhibits the proliferation and promotes apoptosis in colon cancer cells by targeting Wnt/β-catenin signaling pathway" was retracted in 2024. Reason: duplicated images.

**Table 1:** Sequences of primers used for qPCR analysis

Target genes	Primers	Primer sequences
*miR-34b*	F	5′-TCTATTTGCCATCGTCTA-3′
	R	5′-CAGGCAGCTCATTTGGAC-3′
*U6*	F	5′-CTCGCTTCGGCAGCACA-3′
	R	5′-AACGCTTCACGAATTTGCGT-3′
β*-catenin*	F	5′-ATGGCTACTCAAGCTGAC-3′
	R	5′-CAGCACTTTCAGCACTCTGC-3′
*c-Myc*	F	5′-ATGGCCCATTACAAAGCCG-3′
	R	5′-TTTCTGGAGTAGCAGCTCCTAA-3′
*PCNA*	F	5′-CCTGCTGGGATATTAGCTCCA-3′
	R	5′-CAGCGGTAGGTGTCGAAGC-3′
*cyclin D1*	F	5′-GCTGCGAAGTGGAAACCATC-3′
	R	5′-CCTCCTTCTGCACACATTTGAA-3′
*GAPDH*	F	5′-GATTTGGTCGTATTGGGCGC-3′
	R	5′-GCGCCCAATACGACCAAATC-3′

Abbreviation: PCNA, proliferating cell nuclear antigen.

### Cells transfection

Colon cancer Caco-2 cells were seeded in six-well plates overnight at a density of 1 × 10^6^ cells per well, and grown to 80% confluency for transfection. Cells were transfected with miR-34b mimics or control vector (RiboBio, Guangzhou, China) by using Lipofectamine 3000 (Invitrogen, U.S.A.) according to the instructions. The efficiency of transfection was assessed using the quantitative real-time PCR (qRT-PCR) analysis. Cells were collected for further experiments 48 h after transfection.

### Dual-luciferase reporter assay

TargetScan online software (http://www.targetscan.org/) was used to predict the putative target genes of miR-34b. To confirm the targeted relationship between miR-34b and β-catenin, the wild-type (wt) or mutant-type (mut) 3′-UTR of β-catenin were synthesized and cloned into the pMIR-REPORT™ Luciferase miRNA Expression reporter vector (Thermo Fisher Scientific, Inc.). HEK293 cells were co-transfected with the luciferase reporter plasmids as well as miR-34b mimics or control vector by Lipofectamine 2000 (Invitrogen, U.S.A.). After 24 h of transfection, luciferase assays were performed using the Dual-Luciferase Assay system (Promega, U.S.A.). Firefly luciferase activity was normalized to *Renilla* luciferase activity.

The article "MiR-34b inhibits the proliferation and promotes apoptosis in colon cancer cells by targeting Wnt/β-catenin signaling pathway" was retracted in 2024. Reason: duplicated images.

### Cell proliferation assay

Caco-2 cells transfected with miRNA mimics or control vector were seeded into 96-well plates at a rate of 2 × 10^3^ cells/well. Following 24 h transfection, 10 μl of Cell counting kit-8 (CCK-8) solution was added to each well and incubated for 4 h at 37°C. The absorbance at 450 nm was measured using a microplate assay reader (Thermo, Rochester, NY).

### Cell apoptosis assay

Caco-2 cells transfected with miRNA mimics or control vector were seeded into six-well plates at a rate of 1 × 10^6^ cells/well. Apoptosis was evaluated by the annexin V-fluorescein isothiocyanate (FITC) and propidium iodide (PI) staining kit (Nanjing KeyGen, China). Early and late apoptosis cells were analyzed using a flow cytometer (BD Biosciences, Franklin Lakes, NJ, U.S.A.).

### Cell migration assay

Caco-2 cells transfected with miRNA mimics or control vector were seeded into six-well plates at a rate of 1 × 10^6^ cells/well. The monolayers of cells were scratched using a 200-μl pipette tip when the cells reached 100% confluence. Cells were then washed with culture medium to remove cellular debris and allowed to culture again up to 24 h in serum-free medium. Images at 0 and 24 h were captured under an Eclipse Ti-U inverted microscope (Nikon, Kanagawa, Japan).

### Cell invasion assay

Caco-2 cells transfected with miRNA mimics or control vector were seeded into the upper chambers of 24-well plates (Corning Incorporated, Corning, NY, U.S.A., 24-well insert, pore size: 8 mm) at a rate of 3 × 10^4^ cells/well with serum-free medium. Complete medium containing 10% FBS was placed into the lower chambers as a chemoattractant. After 40 h of incubation, the chamber was removed and cells that migrated through the membrane were fixed with 4% formaldehyde for 15 min at 37°C, washed with PBS and stained with Crystal Violet solution for 20 min at 37°C. Images were observed with an Eclipse Ti-U inverted microscope (Nikon, Kanagawa, Japan) and invaded cell number per field was counted by Image-Pro Plus version 6.0.

### Western blot analysis

Total proteins from Caco-2 cells transfected with miRNA mimics or control vector were extracted using RIPA lysis buffer containing PMSF and 1% protease inhibitor (Beyotime, China). The total protein concentrations were determined by BCA protein assay kit (Beyotime, China). Total protein samples (50 µg) were subjected to SDS/polyacrylamide gel electrophoresis and then transferred on to polyvinylidene fluoride membranes. The membranes were blocked with 5% non-fat milk in TBS + Tween 20 (TBST), and incubated at 4°C overnight with the following primary antibodies: c-Myc (Cell Signaling, U.S.A.), Proliferating cell nuclear antigen (PCNA) (Cell Signaling, U.S.A.), cyclin D1 (Santa Cruz, U.S.A.) and anti-β-catenin (Abcam, U.S.A.) antibody. β-actin (Abcam, U.S.A.) was used as the loading control. Horseradish peroxidase–conjugated secondary antibody were incubated for 1 h at room temperature and detected with an enhanced chemiluminscence kit (Beyotime, China). Finally, the expression levels of proteins were determined using Image-Pro Plus 6.0 software.

The article "MiR-34b inhibits the proliferation and promotes apoptosis in colon cancer cells by targeting Wnt/β-catenin signaling pathway" was retracted in 2024. Reason: duplicated images.

### Statistical analysis

Statistical analysis was performed using SPSS 18.0 statistical software. The data are expressed as means ± SEM and one-way analysis of variance (ANOVA) was used to compare the differences among groups. The comparison between two different groups was performed by *t* test and differences were considered statistically significant if *P*<0.05.

## Results

### Expression level of miR-34b was reduced in colon cancer tissue specimens

To investigate the role of miR-34b in colon cancer development, the expression level of miR-34b in 27 pairs of colon cancer tissues and adjacent non-tumor tissues was determined by qRT-PCR. We found that miR-34b expression was significantly reduced in colon cancer tissues when compared with the adjacent non-tumor tissues (Figure 1), indicating that miR-34b may be a potential tumor suppressor in colon cancer progression.

**Figure 1:** MiR-34b expression was down-regulated in human colon cancer tissues when compared with the adjacent non-tumor tissues The expression of miR-34b was detected by qPCR analysis. The data are expressed as means ± SEM. Statistical analysis was performed using Student’s *t* test.

### MiR-34b inhibited proliferation and induced apoptosis of colon cancer cells

To further investigate the biological functions of miR-34b, human colon cancer Caco-2 cells were transfected with miR-34b mimic or miR-34b mimic control vector. Transfection efficiency was assessed using qRT-PCR and the results showed that miR-34b was significantly up-regulated in cells transfected with mimic when compared with cells transfected with control vector (Figure 2A).

**Figure 2:** MiR-34b inhibited proliferation and induced apoptosis in Caco-2 cells (**A**) The expression of miR-34b in cells transfected with miR-34b mimic or control vector. (**B**) CCK-8 analysis of proliferation in cells transfected with miR-34b mimic or control vector at 0, 12, 24 and 48 h. (**C**) Flow cytometry analysis of apoptosis in cells transfected with miR-34b mimic or control vector. *n*=3 per group. The data are expressed as means ± SEM. *P<0.05 and **P<0.01. Statistical analysis was performed using one-way ANOVA followed by Bonferroni’s post hoc test or Student’s *t* test.

We further investigated the effects of miR-34b on proliferation and apoptosis of Caco-2 cells, CCK-8 assay showed that miR-34b overexpression significantly inhibited cell proliferation (*P*<0.05) (Figure 2B). In consistence with this result, flow cytometry showed that overexpression of miR-34b significantly induced cell apoptosis (*P*<0.01) (Figure 2C). These results suggest that miR-34b may inhibit the proliferation of colon cancer cells by inducing apoptosis.

The article "MiR-34b inhibits the proliferation and promotes apoptosis in colon cancer cells by targeting Wnt/β-catenin signaling pathway" was retracted in 2024. Reason: duplicated images.

### MiR-34b inhibits migration and invasion of colon cancer cells

Wound-healing assay and transwell assay were performed to explore the role of miR-34b in regulating cancer cell metastasis. The results showed that the relative migration rate of cells transfected with miR-34b mimic were significantly reduced when compared with cells transfected with control vector (Figure 3A). In addition, overexpression of miR-34b significantly inhibited the number of invasive cells in cells transfected with miR-34b mimic when compared with cells transfected with control vector (*P*<0.001) (Figure 3B). Thus, these results suggest that miR-34b may play important roles in inhibition of colon cancer metastasis.

**Figure 3:** MiR-34b inhibited migration and invasion in Caco-2 cells (**A**) Wound-healing assay of migration in cells transfected with miR-34b mimic or control vector. (**B**) Transwell assay of invasion in cells transfected with miR-34b mimic or control vector. *n*=3 per group. The data are expressed as means ± SEM. ***P<0.001. Statistical analysis was performed using Student’s *t* test.

### β-catenin was directly targeted by miR-34b

To investigate the molecular mechanisms of how miR-34b suppresses colon cancer cell growth, the target mediators of miR-34b were analyzed using TargetScan Website (TargetScan, http://www.targetscan.org). Notably, β-catenin, which has been reported to be associated with miR-34a in colon cancer development [13], may be one potential gene targeted by miR-34b (Figure 4A). We thus examined the expression level of β-catenin in tissues of colon cancer patients. Of note, the expression level of β-catenin was significantly higher in colon cancer tissues when compared with the adjacent non-tumor tissues (Figure 4B).

**Figure 4:** β-catenin was a direct target of miR-34b (**A**) The binding sites between 3′UTR of β-catenin and miR-34b predicted by using TargetScan website. (**B**) The expression of miR-34b in human colon cancer tissues. (**C**) The mRNA and protein expression levels of β-catenin in cells transfected with miR-34b mimic or control vector. (**D**) The luciferase activity in HEK293 cells transfected with miR-34b mimic or control vector combined with wt or mut 3′ UTR sequence of β-catenin. *n*=3 per group. The data are expressed as means ± SEM. *P<0.05 and **P<0.01. Statistical analysis was performed using one-way ANOVA followed by Bonferroni’s post hoc test or Student’s *t* test.

The article "MiR-34b inhibits the proliferation and promotes apoptosis in colon cancer cells by targeting Wnt/β-catenin signaling pathway" was retracted in 2024. Reason: duplicated images.

We further explored the regulatory effects of miR-34b on β-catenin expression. The mRNA levels of β-catenin were measured after 293T cells transfected with miR-34b mimic or control vector. As shown in Figure 4C, the expression of β-catenin at both mRNA and protein levels were significantly inhibited in cells transfected with miR-34b mimic when compared with cells in the control group, suggesting that β-catenin may act as an important target of miR-34b. No study so far investigated the direct interaction between miR-34b and β-catenin in colon cancer cells. To test whether miR-34b directly targeted β-catenin, the wt or mut 3′ UTR sequence of β-catenin was cloned into a luciferase reporter vector. The results revealed that miR-34b significantly reduced the luciferase activity of HEK293 cells when the reporter gene contained the 3′UTR of β-catenin. However, the luciferase response to miR-34b was abrogated when the putative miR-34b binding site in the 3′UTR of β-catenin was mutated (Figure 4D). Therefore, these results illustrate that β-catenin may be a direct target of miR-34b.

### The effects of miR-34b on colon cancer cells was through Wnt/β-Catenin signaling

We then determined the effects of miR-34b on the expression of key mediators in Wnt/β-catenin signaling, which has been reported to be closely associated with colon cancer progression [17]. As shown in Figure 5A,B, overexpression of miR-34b significantly decreased the mRNA and protein expression levels of c-Myc, PCNA and cyclin D1 in Caco-2 cells when compared with cells transfected with control vector. These results suggest that Wnt/β-Catenin signaling pathway may be a key downstream effector in mediating the effects of miR-34b on the colon cancer cells.

**Figure 5:** The effects of miR-34b on Wnt/β-Catenin signaling (**A**) The mRNA expression levels of c-Myc, PCNA and cyclin D1 in cells transfected with miR-34b mimic or control vector. (**B**) Western blot analysis of the protein expression levels of c-Myc, PCNA and cyclin D1 in cells transfected with miR-34b mimic or control vector. *n*=3 per group. The data are expressed as means ± SEM. *P<0.05, **P<0.01 and ***P<0.001. Statistical analysis was performed using Student’s *t* test.

## Discussion

Colon cancer is one of the most common digestive cancers with a relatively high mortality, leading to a huge health burden worldwide [1]. However, the pathogenesis of colon cancer is still unclear. Accumulating evidence has indicated that miRNAs play crucial role in contributing to the carcinogenesis and progression of colon cancer [5,6]. In the present study, the role of miR-34b in regulating the growth, migration, invasion and apoptosis of colon cancer cells as well as the underlying mechanisms were studied.

The article "MiR-34b inhibits the proliferation and promotes apoptosis in colon cancer cells by targeting Wnt/β-catenin signaling pathway" was retracted in 2024. Reason: duplicated images.

MiRNAs are a class of small non-coding RNAs molecules that negatively regulate gene expression through binding to their target mRNAs [18]. It has been reported that abnormal miRNAs expression plays important roles in the initiation, progression and metastasis of several human cancers [5]. The dysregulated expression of several miRNAs, including miR-378 [19], miR-766 [20], miR-21 [21] and miR-136 [22], has been reported to be associated with progression of colon cancer. In the present study, we found that the expression of miR-34b was significantly down-regulated in human colon cancer tissues when compared with adjacent non-tumor tissues, suggesting that miR-34b may play a vital role in the tumorigenesis and progression of human colon cancer. We further investigated the biological functions of miR-34b by performing the ectopic expression of miR-34b in colon cancer cells. We found that overexpression of miR-34b significantly suppressed the proliferation, migration, invasion and induced apoptosis of Caco-2 cells, suggesting that miR-34b may act as a tumor suppressor in colon cancer development. Consistent with our results, previous studies have also demonstrated that miR-34b may serves as a tumor suppressor in other human cancers [23]. For example, down-regulated expression of miR-34b was observed in patients with nasopharyngeal carcinoma and miR-34b overexpression effectively suppressed the growth of nasopharyngeal carcinoma cells by targeting lactate dehydrogenase A [24]. Moreover, overexpression of miR-34b could inhibit proliferation, migration and invasion in prostate cancer cells also by regulating the TGF-β signaling pathway [25]. In addition, by directly targeting YY1-associated factor 2, a recent study demonstrated that miR-34b could inhibit migration and promote apoptosis of lung cancer cells [26]. These findings suggest that miR-34b may be a valuable marker for prognosis of colon cancer and the correlation between miR-34b and the disease status of colon cancer patients should be conducted in our further research.

It is known that miRNAs exert biological functions by inhibiting the expression of target genes [4]. We thus further used bioinformatics program to predict the potential mediators of miR-34b and found that β-catenin was a candidate target for miR-34b. Studies have demonstrated that β-catenin is highly associated with tumorigenesis and plays critical roles in cancer cell proliferation and apoptosis [27,28]. In the present study, luciferase reporter assays identified that β-catenin was a direct target of miR-34b and ectopic expression of miR-34b significantly suppressed mRNA and protein levels of β-catenin in Caco-2 cells. To the best of our knowledge, this is the first study demonstrating that β-catenin is a direct target of miR-34 in human colon cancer cells. Consistent with the results of our findings, a previous study demonstrated that transient overexpression of miR-34b or miR-34c inhibited the expression of endogenous β-catenin in prostate cancer cells [29]. The directly targeted relationship between miR-34 and β-catenin was also observed in human breast cancer MCF-7 cells and lung cancer A549 cells [30]. Thus, our findings indicate that miR-34b may inhibit proliferation and promote apoptosis in human colon cancer cells, at least in part, via directly suppressing β-catenin expression.

β-catenin is also the central and most well-studied signaling molecule in the Wnt pathway [31]. Wnt/β-catenin signaling is a critical pathway for regulating cell growth and differentiation and aberrant activation of Wnt/β-catenin signaling pathway has been frequently identified in many tumor types, such as breast cancer [32], liver cancer [33], prostate cancer [34] and colon cancer [35]. We thus further examined the expression of key Wnt/β-catenin signaling mediators in cells transfected with miR-34b mimic and cells transfected with control vector. It has been demonstrated that c-Myc, PCNA and cyclin D1 are key signatory genes of Wnt signaling [36]. Oncoprotein c-MYC is overexpressed in many human cancers and is a transcription factor that involved in the regulation of many cellular processes such as cell cycle, survival and metabolism [37,38]. PCNA a non-histamine nuclear protein that has been described as a biomarker of colorectal adenocarcinoma [39]. Moreover, Cyclin D1 is a regulator that responsible for cell cycle progression and has also been associated with tumor invasion and metastasis in many clinical studies [40]. In this study, we demonstrated that miR-34b overexpression significantly decreased the protein expression levels of c-MYC, PCNA and Cyclin D1 in Caco-2 cells, indicating that Wnt/β-Catenin is a key downstream signaling pathway in response to the regulation of miR-34b in colon cancer cells. It should be noted that Runx is also an important transcription factor associated with Wnt/β-Catenin signaling pathway in cancer development [41–43], further studies are needed to investigate whether there is a close relationship between miR-34b and Runx.

The article "MiR-34b inhibits the proliferation and promotes apoptosis in colon cancer cells by targeting Wnt/β-catenin signaling pathway" was retracted in 2024. Reason: duplicated images.

In conclusion, the expression of miR-34b was significantly down-regulated in human colon cancer samples and overexpression of miR-34b effectively inhibited the proliferation and promoted apoptosis in colon caner cells possibly through regulating the Wnt/β-catenin signaling pathway. Thus, our findings suggest that miR-34b may serve as a potential therapeutic candidate in the treatment of colon cancer.

## Abbreviations

CCK-8: cell counting kit-8
miRNA: microRNA
mut: mutant
PCNA: proliferating cell nuclear antigen
qRT-PCR: quantitative real-time PCR
wt: wild-type
